RETRACTED

# Circulating MicroRNAs as a Novel Class of Diagnostic Biomarkers in Gastrointestinal Tumors Detection: A Meta-Analysis Based on 42 Articles

**DOI:** 10.1371/journal.pone.0113401

**Published:** 2014-11-18

**Authors:** Ran Wang, Hong Wen, Yongcheng Xu, Qiulan Chen, Yi Luo, Yiqin Lin, Yu Luo, Angao Xu

**Affiliations:** 1 Department of Gastroenterology, Nanfang Hospital, Southern Medical University, Guangzhou, China; 2 Department of Ultrasound, HuiZhou Municipal Central Hospital, Huizhou, China; 3 Department of Gastroenterology, HuiZhou Municipal Central Hospital, Huizhou, China; Geisel School of Medicine at Dartmouth College, United States of America

## Abstract

**Objective:**

MicroRNAs (miRNAs) have become the focus of most recent efforts in cancer research. However, there have been inconsistencies in the literature regarding the suitability of circulating miRNAs for early detection of gastrointestinal cancers. This study aims to assess the diagnostic performance of circulating miRNAs in detection of gastrointestinal cancer through a meta-analysis.

**Methods:**

Eligible studies were selected by conducting a systematic literature search of public databases. The sensitivity and specificity were used to plot the summary receiver operator characteristic (SROC) curve and calculate the area under the SROC curve (AUC). The between-study heterogeneity was evaluated by *Q* test and *I* ^2^ statistics. Subgroup analyses and meta-regression were further performed to explore the potential sources of heterogeneity. All analyses were performed using the STATA 12.0 software.

**Results:**

A total of 107 studies from 42 articles were included for the meta-analysis according to the inclusion criteria. The overall analysis of all gastrointestinal cancers showed that circulating miRNAs have a relatively good diagnostic performance in gastrointestinal cancers, with a sensitivity of 0.75, a specificity of 0.81 and an AUC of 0.85. In addition, subgroup analyses based on different type of miRNA assay suggested that single-miRNA assay displayed a relatively low diagnostic performance with the AUC values of 0.84 for gastric cancer (GC) and 0.79 for colorectal cancer (CRC), while multiple-miRNAs assay significantly improved the diagnosing accuracy with AUC rising to 0.92 for GC and 0.89 for CRC. Another interesting finding was that plasma-based miRNA assay reach a higher accuracy compared with serum-based one for GC, while opposite conclusion was drawn for CRC.

**Conclusions:**

In conclusion, circulating miRNAs, particularly the combination of multiple miRNAs, may present as promising biomarkers for the diagnosis of gastrointestinal cancers. Further large-scale prospective studies are necessary to validate their potential applicability in human cancer diagnosis.

RETRACTED

## Introduction

Gastrointestinal tract cancers, especially gastric, colorectal, and esophageal cancers, are one of the most common causes of cancer-related deaths [1]. It was estimated that tumors in esophagus, stomach, and colorectum account for approximately 11% of all newly diagnosed cancers and 14% of cancer related deaths in the United States in 2013, which make it an epidemiological health concern [2]. Currently, one of the biggest challenges in cancer treatment is the lack of specific and sensitive biomarker for early cancer diagnosis, which hinders the patients from receiving the timely treatment. The 5-year survival rate after surgical resection reaches 90% for gastric cancer (GC) patients at stage I, but this rate dramatically drops to 5% in cases at stage IV [3]. For colorectal cancer (CRC) patients, the 5-year survival rate of stage II cases is over 80% after surgical resection, but less than 10% at advanced [4]. In addition, the locoregional recurrence and/or distant metastasis can be frequently observed in the late-stage cancer patients even if they have already received the resection and multimodality therapy [5]. Therefore, the low survival rate of cancer patients at advanced stages highlights the importance of early cancer diagnosis. Unfortunately, most human cancers show no symptom in at early stages, which makes it hard for early diagnosis, and the cost-effectiveness of available diagnostic techniques is unsatisfactory.

Currently, the wide range of conventional diagnostic methods, including gastroscopy, random biopsies, colonoscopy, double contrast barium enema (DCBE), and computed tomographic colonography (CTC), are applied to diagnose and monitor gastrointestinal cancers. Although gastroscopy/colonoscopy is currently considered to be the most reliable screening tool with reportedly high accuracy, its invasive nature and expensive cost have hindered its widespread application in cancer diagnosis as a screening tool [6], [7]. DCBE and CTC can detect some intestinal cancers at an early stage, but the complicated diagnostic procedures as well as the associated radiation hazards also limit their clinical applications [8]. In addition, fecal-based analyses, such as occult blood and stool DNA tests, are currently most common non-invasive procedure for early cancer diagnosis [9], [10]. However, the lack of sufficient sensitivity and specificity hampers their utility in the detection of premalignant lesions.

It is generally believed that cancer-related biomarkers in blood would be quite helpful in early cancer diagnosis and tumor progression monitoring. Several currently available circulating biomarkers, such as carbohydrate antigen 19-9 (CA 19-9), carcinoembryonic antigen (CEA), pepsinogen (PG) I/II ratio, estrogen receptor (ER), and progesterone receptor (PR), are being used as non-invasive methods for cancer diagnosis without involving a biopsy or a surgical procedure [11]–[13]; Unfortunately, they also suffer from the limitation of low sensitivities and specificities. Therefore, there is a pressing need for novel and more sensitive non-invasive biomarkers to improve the diagnostic accuracy for gastrointestinal cancers.

RETRACTED

Recently, circulating miRNAs have attracted considerable attention in its diagnostic value for human cancers. MiRNAs are a family of small non-coding functional RNAs with 19–24 nucleotides modulating the expression of messenger RNA (mRNA) [14]. In recent years, miRNAs have been found to be dysregulated in a variety of diseases, particularly in human cancers [15], [16]. It has been observed that miRNAs could present extensively in the cell-free body fluids and excretions, including serum, plasma, urine, tears, saliva, bronchial lavage, and feces, etc [17]. Furthermore, biochemical analyses indicate that circulating miRNAs have a remarkable stability and are tolerant to RNase activity and extreme physiological environment [18], making it plausible to use circulating miRNAs as novel non-invasive biomarkers in diagnosing and monitoring human cancers.

The role of miRNAs as novel biomarkers in cancer was first recognized in a study considering miR-15 and miR-16, which were found to be down-regulated in B-cell chronic lymphocytic leukemia (B-CLL) [19]. Subsequent evidence has indicated that unique miRNA expression profiles in circulation may contribute to the diagnosis of cancers, such as colorectal cancer [20], gastric cancer [21], esophageal cancer [22], breast cancer [23], lung cancer [24], hepatocellular carcinoma [25], prostate cancer [26], and pancreatic cancer [27]. However, there have been inconsistencies or discrepancies in the literature reviews regarding the reliability of circulating miRNAs for early detection of gastrointestinal cancers. In this meta-analysis, we summarize an overview of circulating miRNAs present in blood circulation to further elucidate their diagnostic performance and provide information for the early detection of gastrointestinal cancers.

## Materials and Methods

This meta-analysis was conducted according to the Preferred Reporting Items for Systematic Reviews and Meta-analyses (PRISMA) guidance (Supplement S1).

### Literature search

This meta-analysis was conducted according to guidelines for diagnostic meta-analysis [28]. Eligible studies published up to 1 April 2014 were selected for meta-analysis by conducting a systematic literature search of public databases including PubMed, Embase, Chinese National Knowledge Infrastructure (CNKI), and Chinese Biology Medicine (CBM) databases, without language limitation. The following retrieval strategy was used: (‘gastrointestinal tumor’ OR ‘gastric tumor’ OR ‘gastric cancer’ OR ‘colorectal tumor’ OR ‘colorectal cancer’ OR ‘esophageal tumor’ OR ‘esophageal cancer’) AND (‘microRNA’ OR ‘miRNA’ OR ‘miR’) AND (‘blood’ OR ‘serum’ OR ‘plasma’ or ‘circulating’) AND (‘diagnosis’ OR ‘sensitivity and specificity’ OR ‘ROC curve’). In addition, reference lists of eligible articles were independently searched manually to obtain additional sources.

RETRACTED

### Inclusion and exclusion criteria

Eligible studies included in this meta-analysis have to fulfill the following criteria: (1) studies regarding the diagnostic potential of circulating miRNAs for gastrointestinal cancers; (2) studies with a gold reference standard for the gastrointestinal cancers diagnosis; (3) studies with sufficient data for construction of two-by-two tables [i.e., true positive (TP), false positive (FP), true negative (TN) and false negative (FN)]. Exclusion criteria were: (1) publications unrelated to the diagnostic values of circulating miRNAs for gastrointestinal cancers; (2) studies with duplicate data reported in other studies; (3) letters, editorials, case reports or reviews.

### Data extraction

Two reviewers independently extracted data from all the eligible studies: (1) basic characteristics of studies, including name of the first author, year of publication, country of origin, ethnicity, study design, sample size, mean age, male ratio, cancer type, type of miRNA assay, methods of miRNAs detection, type of specimens; and (2) diagnostic performance, including sensitivity, specificity, TP, FP, FN, and TN.

### Quality assessment

The qualities of included studies were scored independently by two reviewers using the revised Quality Assessment of Diagnostic Accuracy Studies (QUADAS-2) criteria [29]. The QUADAS-2 tool is comprised of 4 key domains: patient selection, index test, reference standard and flow and timing, and uses seven questions to evaluate the quality of included studies (Supplements S2). Each question is answered with “yes”, “no”, or “unclear”. An answer of “yes” means that the risk of bias can be judged low, while an answer of “no” or “unclear” means that the risk of bias can be judged high. In case of conflict, a third reviewer was consulted, and disagreement was settled through multilateral discussion.

### Statistical analysis

All analyses were performed using the STATA 12.0 software. The bivariate meta-analysis model was employed to summarize the sensitivity (SEN), specificity (SPE), positive likelihood ratio (PLR), negative likelihood ratio (NLR) and diagnostic odds ratio (DOR) [30], [31]. The sensitivity and specificity of each included study were used to plot the summary receiver operator characteristic (SROC) curve and calculate the area under the SROC curve (AUC). The AUC can be statistically interpreted as the probability to correctly distinguish patients from normal controls. The between-study heterogeneity was evaluated by *Q* test and *I* ^2^ statistics. A *P* value less than 0.10 for *Q* test or *I* ^2^ values ≥50% indicates substantial heterogeneity, and then the random-effects model was applied [32], [33]. To further explore the potential sources of heterogeneity, subgroup analyses and meta-regression were performed according to the characteristics of the included studies. As publication bias is a concern for meta-analyses, Deeks' funnel plot asymmetry test was used, with *P*<0.10 indicating statistically significant [34].

RETRACTED

## Results

### Procedure of literature retrieval

The procedure of the literature retrieval was presented in Figure 1. The initial search returned a total of 301 articles, of which 13 duplicate publications among databases were removed. After the review of titles and abstracts, 206 articles were excluded: 56 were reviews or letters, 23 were not human studies, and 127 were not related to our research topic, leaving 82 articles available for further full-text review. After careful reading, 40 articles were further excluded: 20 were not about gastrointestinal cancers diagnosis, 3 were relevant to metastasis in cancers, and 17 were not circulating miRNAs. Finally, 42 articles were included according to the inclusion criteria, 21 of which focused on GC [21], [35]–[54], 15 on CRC [20], [49], [55]–[67], and the other 6 on EC [22], [68]–[72].

**Figure 1:** Flow diagram of study selection process.

### Baseline characteristics of included studies

The main characteristics of 42 articles were shown in Table 1. In total, 107 studies from these 42 articles were involved in the current meta-analysis. As for GC, 47 studies from 21 articles were available for analysis. 38 of these 47 studies investigated the diagnostic value of single-miRNA assay in GC detection, while only 8 focused on multiple-miRNAs assay. 26 studies used plasma as specimen, and the other 21 based on serum. Similarly, for 47 studies from the 15 articles focusing on CRC, 29 of them assessed the performance of single-miRNA assay in CRC detection, whereas 18 focused on multiple-miRNAs assay. 33 studies used plasma as specimen, while serum was applied in the other 14 studies. For EC diagnosis, 13 studies from 6 articles were available. The publication years of the included articles range from 2010 to 2014. All studies used the quantitative real-time reverse transcription-PCR (qRT-PCR) method to measure the expression of circulating miRNAs. Quality assessment for the overall studies was shown with a bar graph according to the QUADAS-2 tool in Figure 2. The majority of all included studies in this meta-analysis fulfilled 4 or more of the 7 items in QUADAS-2, indicating that the overall quality of included studies is generally good.

RETRACTED

**Figure 2:** Overall quality assessment of included studies using the QUADAS-2 criteria (a: risk of bias; b: applicability).

**Table 1:** Main characteristics of 42 studies included in meta-analysis.

Included studies	Cancer type	Location	Ethnicity	Study design	Case/Control			miRNA profiling	Specimen	QUADAS
					Number	Mean age	Male ratio			
Cai H, 2013	GC	China	Asian	Case-control	90/90	46.2/46.1	0.81/0.81	miR-106b, -20a, -221	Plasma	5
Chen Q, 2014	GC	China	Asian	Case-control	36/36	56/59	0.78/0.78	miR-122, -192	Plasma	6
Konishi H, 2012	GC	Japan	Asian	Case-control	56/30	66/NA	0.55/NA	miR-451, -486	Plasma	7
Li BS, 2012	GC	China	Asian	Case-control	60/60	54/51	0.70/0.63	miR-223, -21, -218	Plasma	4
Li C, 2013	GC	China	Asian	Case-control	180/80	58.1/58.9	0.31/0.35	miR-199a-3p, -151-5p	Plasma	5
Li ZQ, 2012	GC	China	Asian	Case-control	46/21	58.8/57	0.65/0.67	miR-27a, -181b	Plasma	5
Liu H, 2012	GC	China	Asian	Case-control	40/41	56/58	0.66/0.66	miR-371-5p, -187, -378	Serum	3
Liu R, 2011	GC	China	Asian	Case-control	164/127	60.2/60	0.84/0.8	miR-1, -20a, -27a, -34, -423-5p	Serum	4
Peng WZ, 2014	GC	China	Asian	Case-control	57/58	NA/43	NA/0.48	miR-191, -425	Serum	5
Sheinerman KS, 2013	GC	America	Caucasian	Case-control	10/30	55.8/51.9	0.10/0.30	miR-203, -146b-5p, -192	Plasma	6
Shiotani A, 2013	GC	Japan	Asian	Case-control	64/64	67.9/68.4	0.70/0.64	miR-106b, let-7	Serum	5
Song MY, 2012	GC	China	Asian	Retrospective	68/68	60.4/60.4	0.71/0.71	7 miRNAs^a^	Serum	4
Tsujiura M, 2010	GC	Japan	Asian	Case-control	69/30	NA/NA	NA/NA	miR-106b	Plasma	5
Valladares M, 2012	GC	Spain	Caucasian	Case-control	52/15	65.9/65.3	0.81/0.81	miR-200c	Plasma	7
Wang B, 2012	GC	China	Asian	Case-control	30/39	58/46	0.73/0.77	miR-21	Serum	3
Xu Q, 2013	GC	China	Asian	Case-control	94/103	60.2/59.1	0.63/0.63	miR-320a	Serum	4
Zheng Y, 2011	GC	China	Asian	Case-control	53/20	60/60	0.66/0.66	miR-21	Serum	4
Zhou H, 2010	GC	China	Asian	Case-control	90/27	62.3/NA	0.70/NA	miR-106a, -17	Serum	4
Zhou H, 2012	GC	China	Asian	Case-control	40/17	64.6/64.6	0.73/0.73	miR-421	Serum	4
Zhu C, 2014	GC	China	Asian	Case-control	40/40	53.8/53.5	0.73/0.73	miR-16, -25, -92a, -451, -468-5p	Plasma	3
Zhu CJ, 2011	GC	China	Asian	Case-control	48/27	61.2/55.4	0.83/0.74	miR-191, -27a	Plasma	6
Feng L, 2013	CRC	China	Asian	Case-control	98/50	54.3/52.7	0.53/0.52	miR-92a	Serum	7
Giraldez MD, 2013	CRC	Spain	Caucasian	Cohort	42/53	62.8/62.1	0.51/0.49	miR-19a, -19b, -15b	Plasma	4
Huang Z, 2010	CRC	China	Asian	Case-control	100/59	61/58	0.51/0.53	miR-29a, -92a	Plasma	3
Liu et al, 2013	CRC	China	Asian	Cohort	200/80	57.9/57.5	0.63/0.52	miR-21, 92a	Serum	6
Liu HS, 2012	CRC	China	Asian	Case-control	47/28	58.6/56.2	0.66/0.68	miR-129-3p, -767-3p, -877	Serum	4
Luo X, 2013	CRC	Germany	Caucasian	Case-control	80/144	68/62.5	0.56/0.42	12 miRNAs^b^	Plasma	5
Ng EK, 2009	CRC	China	Asian	Case-control	90/50	71/69	0.52/0.52	miR-17-3p, -92	Plasma	5
Pu XX, 2010	CRC	China	Asian	Cohort	103/37	58/32	0.64/0.51	miR-221	Plasma	7
Sheinerman KS, 2013	CRC	America	Caucasian	Case-control	10/30	57.8/57.3	0.80/0.30	miR-203, -146b-5p, -192, -215, -303-3p	Plasma	3
Toiyama Y, 2013	CRC	Japan	Asian	Cohort	186/53	67.5/64	0.57/0.51	miR-21	Serum	3
Wang Q, 2012	CRC	China	Asian	Case-control	90/58	62/58	0.50/0.52	miR-601, -760, -29a, -92a	Plasma	6
Wang S, 2013	CRC	China	Asian	Cohort	77/84	64/44	0.42/0.60	miR-409-3p, -7, -93	Plasma	4
Yong FL, 2013	CRC	Malaysia	Asian	Case-control	70/32	64.4/61.5	0.60/0.48	miR-193a-3p, -23a, -338-5p	Serum	5
Zanutto S, 2014	CRC	Italy	Caucasian	Cohort	29/29	NA/NA	NA/NA	miR-378, -21	Plasma	5
Zhang GJ, 2013	CRC	China	Asian	Case-control	78/86	61.4/60.3	0.55/0.62	miR-200c, 18a	Plasma	4
Hirajima S, 2013	EC	Japan	Asian	Case-control	106/54	65/NA	0.82/NA	miR-18a	Plasma	5
Komatsu S, 2011	EC	Japan	Asian	Case-control	50/20	65/NA	0.88/NA	miR-21/-375	Plasma	7
Takeshita N, 2013	EC	Japan	Asian	Case-control	101/46	NA/NA	0.89/NA	miR-1246	Serum	3
Zhang C, 2010	EC	China	Asian	Cohort	149/100	62/50	0.78/0.74	7 miRNAs^c^	Serum	4
Zhang T, 2011	EC	China	Asian	Cohort	201/202	NA/NA	0.66/0.63	miR-31	Serum	3
Zhang T, 2013	EC	China	Asian	Case-control	201/201	NA/NA	0.66/0.62	miR-1322	Serum	6

a miR-221, -744, -376c, -27a, -27b, -222, -191.

b miR-18a, -20a, -21, -29a, -92a, -106b, -133a, -143, -145, -181b, -342-3p, -532-3p.

c miR-10a, -22, -100, -148b, -223, -133a, -127-3p.

RETRACTED

NA, not available; GC, gastric cancer; CRC, colorectal cancer; EC, esophageal cancer; QUADAS-2, the revised Quality Assessment of Diagnostic Accuracy Studies.

### Diagnostic accuracy of miRNAs in gastrointestinal cancers

The pooled estimates of gastrointestinal cancers (GC/CRC/EC) for the diagnostic accuracy of circulating miRNAs were presented in Table 2. The overall analysis of all types gastrointestinal cancers showed that circulating miRNAs have a relatively good diagnostic performance in gastrointestinal cancers, with SEN of 0.75 (95% CI: 0.73–0.78), SPE of 0.81 (95% CI: 0.79–0.83) and AUC of 0.85 (95% CI: 0.82–0.88) (Figure 3A). Since only 13 studies from 6 publications were involved in EC, subgroup analyses were conducted for GC and CRC. For EC, the diagnostic accuracy of circulating miRNAs was even better than the overall results, with SEN of 0.79 (95% CI: 0.74–0.84), SPE of 0.85 (95% CI: 0.81–0.89) and AUC of 0.89 (95% CI: 0.86–0.92) (Figure 3D).

**Figure 3:** SROC curve with pooled estimates of sensitivity, specificity and AUC (a: overall studies on gastrointestinal cancers; b: GC; c: CRC; d: EC).

**Table 2:** Summary estimates of diagnostic criteria and their 95% confidence intervals (95% CI).

Analysis	No. of studies	SEN (95%CI)	SPE (95%CI)	PLR (95%CI)	NLR (95%CI)	DOR (95%CI)	AUC (95%CI)
**Gastric cancer**	47	0.77 (0.72–0.80)	0.81 (0.77–0.84)	4.0 (3.2–4.9)	0.29 (0.24–0.36)	14 (9–20)	0.86 (0.82–0.88)
MiRNA profiling							
Single-miRNA	39	0.75 (0.70–0.79)	0.80 (0.75–0.84)	3.7 (2.9–4.6)	0.32 (0.26–0.39)	11 (8–17)	0.84 (0.80–0.87)
Multiple-miRNAs	8	0.87 (0.75–0.94)	0.84 (0.75–0.91)	5.6 (3.1–10)	0.15 (0.07–0.33)	37 (10–134)	0.92 (0.89–0.94)
Source material							
Plasma-based	26	0.82 (0.78–0.86)	0.85 (0.80–0.89)	5.6 (4.0–7.8)	0.21 (0.16–0.27)	27 (16–47)	0.90 (0.88–0.93)
Serum-based	21	0.67 (0.61–0.73)	0.74 (0.69–0.78)	2.5 (2.1–3.1)	0.44 (0.37–0.53)	6 (4–8)	0.77 (0.73–0.80)
**Colorectal cancer**	47	0.73 (0.69–0.77)	0.80 (0.76–0.83)	3.6 (3.0–4.2)	0.34 (0.29–0.39)	11 (8–14)	0.83 (0.80–0.86)
MiRNA profiling							
Single-miRNA	29	0.68 (0.62–0.73)	0.77 (0.72–0.81)	2.9 (2.4–3.5)	0.42 (0.36–0.50)	7 (5–10)	0.79 (0.75–0.82)
Multiple-miRNAs	18	0.81 (0.77–0.84)	0.83 (0.79–0.87)	4.9 (3.8–6.2)	0.23 (0.19–0.27)	22 (15–30)	0.89 (0.86–0.91)
Source material							
Plasma-based	33	0.72 (0.65–0.77)	0.77 (0.73–0.80)	3.1 (2.5–3.7)	0.37 (0.30–0.46)	8 (6–12)	0.81 (0.77–0.84)
Serum-based	14	0.77 (0.72–0.81)	0.85 (0.80–0.89)	5.1 (3.9–6.7)	0.28 (0.23–0.33)	18 (13–26)	0.88 (0.85–0.90)
**Esophageal cancer**	13	0.79 (0.74–0.84)	0.85 (0.81–0.89)	5.4 (4.1–7.1)	0.24 (0.19–0.31)	22 (14–35)	0.89 (0.86–0.92)
**All studies**	107	0.75 (0.73–0.78)	0.81 (0.79–0.83)	4.0 (3.5–4.5)	0.30 (0.27–0.34)	13 (10–16)	0.85 (0.82–0.88)

CI, confidence interval; SEN, sensitivity; SPE, specificity; PLR, positive likelihood ratio; NLR, negative likelihood ratio; DOR, diagnostic odds ratio; AUC, area under the curve.

As for GC, since significant heterogeneity between studies was observed in sensitivity and specificity data (*I* ^2^ = 84.53% and *I* ^2^ = 78.98%, respectively), the random-effects model was used. The pooled parameters calculated from all 47 studies on GC were as follows: SEN, 0.77 (95% CI: 0.72–0.80); SPE, 0.81 (95% CI: 0.77–0.84); PLR, 4.0 (95% CI: 3.2–4.9); NLR, 0.29 (95% CI: 0.24–0.36); and DOR, 14 (95% CI: 9–20). Figure 3B shows the corresponding SROC curve with the AUC of 0.86 (95%CI: 0.82–0.88), indicating that circulating miRNAs may be able to differentiate GC patients from controls with a relatively high accuracy. Subgroup analysis based on different type of miRNA assay suggested that multiple-miRNAs assay showed superior diagnostic properties (Figure 4B) than single one (Figure 4A), with SEN of 0.87 versus 0.75, SPE of 0.84 versus 0.80, and AUC of 0.92 versus 0.84 (Table 2). Notably, we found that plasma-based assay (Figure 4C) has a higher accuracy compared with serum-based assay (Figure 4D), suggesting that plasma is a better matrix for miRNA detection.

RETRACTED

**Figure 4:** SROC curve with pooled estimates of sensitivity, specificity and AUC on the diagnostic value of circulating miRNAs in GC detection (a: single-miRNA assay; b: multiple-miRNAs assay; c: plasma-based assay; d: serum-based assay).

Similarly, the random-effects model was used for meta-analysis of studies on CRC since significant heterogeneity existed (*I* ^2^ = 87.18% and *I* ^2^ = 83.27%, respectively). The pooled estimates all 47 studies on CRC are as follows: SEN of 0.73 (95% CI: 0.69–0.77), SPE of 0.80 (95% CI: 0.76–0.83), PLR of 3.6 (95% CI: 3.0–4.2), NLR of 0.34 (95% CI: 0.29–0.39), and DOR of 11 (95% CI: 8–14) (Table 2). Figure 3C shows the corresponding SROC curve with the AUC of 0.83 (95%CI: 0.80–0.86), indicating that the diagnostic accuracy of miRNAs in CRC detection is slightly worse than the overall diagnostic performance of miRNAs in gastrointestinal cancers detection. Similar to miRNAs in GC detection, we found that multiple-miRNAs assay (Figure 5B) in differentiating CRC patients from controls achieve a better diagnostic performance than single-miRNA assay (Figure 5A). However, contrast to the results of GC, serum-based miRNAs assay (Figure 5D) has a higher accuracy compared with plasma-based assay (Figure 5C) in CRC detection.

**Figure 5:** SROC curve with pooled estimates of sensitivity, specificity and AUC on the diagnostic value of circulating miRNAs in CRC detection (a: single-miRNA assay; b: multiple-miRNAs assay; c: plasma-based assay; d: serum-based assay).

### Meta-regression and publication bias

The meta-regression analyses for both GC (Figure 6A) and CRC (Figure 6B) were performed to analyze the potential sources of inter-study heterogeneity. Overall, miRNA profiling and sample types may be the major sources of heterogeneity for miRNAs assay either in GC or CRC detection. To assess publication bias of included studies, the Deeks' funnel plot asymmetry test was conducted (Figure 7). As shown in Figure 7, the slope coefficient was associated with a *P*-value of 0.38 for GC, 0.41 for CRC, 0.78 for EC, suggesting a low likelihood of publication bias in our meta-analysis.

RETRACTED

**Figure 6:** Forest plots of multivariable meta-regression analyses for sensitivity and specificity (a: single-miRNA assay; b: multiple-miRNAs assay).

**Figure 7:** The Deeks' test of the diagnostic meta-analysis (a: Deeks' funnel for GC; b: Deeks' funnel for CRC; c: Deeks' funnel for EC. The dotted line indicates the regression line. No publication bias was detected for this meta-analysis (GC: *P* = 0.38; CRC: *P* = 0.41; EC: *P* = 0.78).

## Discussion

Gastrointestinal cancers, including esophageal, gastric, and colorectal cancer, together with breast and lung tumors, are responsible for the most cancer-related mortality [1]. Although endoscopic examinations and random biopsies are currently the most reliable screening tool for gastrointestinal cancers, their invasive, unpleasant, and inconvenient nature as well as potential sampling errors have hampered the wide clinic application. Conventional cancer-specific biomarkers are sufficiently simple and fast; unfortunately, their diagnostic performances have mostly been insufficient for application as a primary tool in population-based screening. Therefore, large number of studies on the search for ideal candidate biomarkers of tumors is still ongoing. During the past few years, miRNAs have become the focus of most recent efforts in cancer research. Since their discovery, emerging evidences suggest that the miRNAs may play important role in tumor suppressing, since the aberrant expression of miRNA was discovered between cancer patients and healthy controls [73], [74]. Subsequently, miRNAs as molecular markers have attracted much attention in cancer diagnosis [20], [21], [44], [54], [67].

Circulating miRNAs, also known as cell-free miRNAs, have a promising future as a novel class of reliable minimally invasive biomarkers for early cancer diagnosis due to their remarkable stability, relatively easy detection, and convenience to measure its sensitivity and specificity [73]. Since circulating miRNAs in serum was first reported [75], a tremendous growth of interest is attracted to the feasibility of circulating miRNAs as potential biomarkers in gastrointestinal malignancies diagnosis. However, inconsistencies are still existed in the literature reviews regarding the reliability of circulating miRNAs for early detection of gastrointestinal cancers. The variations and discrepancies in individual studies are possibly due to their small sample sizes, variations in miRNA assay, and different type of cancers. In this meta-analysis, we summarize the recent findings focusing on the potential of circulating miRNAs as diagnostic biomarkers in gastrointestinal tumors, including esophageal, gastric, and colorectal cancer.

RETRACTED

To the best of our knowledge, this is the first evidence-based meta-analysis to evaluate the diagnostic value of circulating miRNA on gastrointestinal malignancies. The pooled results based on all included studies showed circulating miRNAs yielding an AUC of 0.85 with 75% sensitivity and 81% specificity in discriminating gastrointestinal cancer patients from controls. Although the origin and function of circulating miRNAs in cancer diagnosis have not been systematically elucidated, they have displayed a superior diagnostic performance compared with conventional blood biomarkers like CEA (AUC of 0.549) for EC and CA19-9 for GC (AUC of 0.60). Accordingly, further studies are required to elucidate the mechanism and target of miRNAs and their roles in cellular and molecular pathways. Interestingly, our results suggest that plasma-based miRNA assay reaches a higher accuracy than serum-based one for GC; the conclusion is, however, opposite for CRC. The origin of source-related difference is still unclear and might be explained by unknown mechanism. Thus, large scale investigations are needed in the following study to determine whether the source-related differences truly exist.

Another interesting finding of our study is that single-miRNA assay displayed a relatively low diagnostic performance with the AUC values of 0.84 for gastric cancer (GC) and 0.79 for colorectal cancer (CRC), while multiple-miRNAs assay significantly improved the diagnosing accuracy with AUC rising to 0.92 for GC and 0.89 for CRC, implying that the advantage of using combination of miRNAs to obtain a complete picture. It is widely accepted that using single tumor-related miRNA as disease fingerprints is much simpler and more straightforward than comprehensively detecting panels of miRNAs, but the specificity of biomarkers based on single miRNA is relatively poor. The molecular basis for the limitation of single miRNA as a tumor biomarker is that aberrant levels of single miRNA might be associated with several different types of cancers [76]. Furthermore, cancer develops can be regarded as a result of complex multi-stage process of epigenetic and genomic abnormalities, and thus, should be targeted by multiple miRNAs [77]. Accordingly, employing panels of miRNAs instead of an individual miRNA as biomarkers represents a rational option to circumvent the limitations in utilizing miRNAs as a non-invasive blood-based biomarker in cancer detection, especially for the localized pathological conditions, where regular biopsies are hard to get.

RETRACTED

Although circulating miRNAs have a promising potential as relevant novel non-invasive cancer biomarkers in future as shown in the current study, several limitations need to be addressed. First, methodologies for an accurate absolute quantification of miRNAs suffer from a lack of convention, which limits the cross-comparison between studies performed by different laboratories. Standardized protocol, which should be preferably followed across all studies, needs to be established aiming to minimize protocol-based bias. In addition, some researchers have showed correlations of grade and stage of cancers with specific circulating miRNAs. Therefore, further studies addressing the relationships between miRNAs expression and clinical/pathological parameters are very important and desirable. Third, most included studies in this meta-analysis only distinguished the cancer patients from healthy controls. It is vital to identify and develop panels of miRNAs that can distinguish cancer from other diseases, especially from those with similar symptom diseases. Last but not least, as shown in Table 1, most of included studies were on Asian and little bit on Caucasian/African populations. Therefore, further studies on Caucasian/African populations may be needed.

Based on recent observations in gastrointestinal cancer, we conclude that circulating miRNAs, particularly the combination of multiple-miRNAs, may present as promising minimally invasive approach for the diagnosis and monitoring of gastrointestinal tumors. Further large-scale prospective studies are necessary to validate their potential applicability in human cancer diagnosis.

## Supporting Information

Supplement S1 **PRISMA Checklist.**
(DOC)

Supplement S2 **QUADAS-2 Checklist.**
(PDF)
